# Genome-Wide Identification and Expression Analysis of WRKY Gene Family in *Capsicum annuum* L.

This article has been retracted.

**DOI:** 10.3389/fpls.2016.00211

**Published:** 2016-02-23

**Authors:** Wei-Ping Diao, John C. Snyder, Shu-Bin Wang, Jin-Bing Liu, Bao-Gui Pan, Guang-Jun Guo, Ge Wei

**Affiliations:** ^1^Institute of Vegetable Crops, Jiangsu Academy of Agricultural SciencesNanjing, China; ^2^Jiangsu Key Laboratory for Horticultural Crop Genetic ImprovementNanjing, China; ^3^College of Agricultural, Food and Environment, University of KentuckyLexington, KY, USA

**Keywords:** transcriptional factor, WRKY, phylogenetics analysis, expression pattern, pepper

## Abstract

The WRKY family of transcription factors is one of the most important families of plant transcriptional regulators with members regulating multiple biological processes, especially in regulating defense against biotic and abiotic stresses. However, little information is available about WRKYs in pepper (*Capsicum annuum* L.). The recent release of completely assembled genome sequences of pepper allowed us to perform a genome-wide investigation for pepper WRKY proteins. In the present study, a total of 71 WRKY genes were identified in the pepper genome. According to structural features of their encoded proteins, the pepper WRKY genes (*CaWRKY*) were classified into three main groups, with the second group further divided into five subgroups. Genome mapping analysis revealed that *CaWRKY* were enriched on four chromosomes, especially on chromosome 1, and 15.5% of the family members were tandemly duplicated genes. A phylogenetic tree was constructed depending on WRKY domain' sequences derived from pepper and *Arabidopsis*. The expression of 21 selected *CaWRKY* genes in response to seven different biotic and abiotic stresses (salt, heat shock, drought, *Phytophtora capsici*, SA, MeJA, and ABA) was evaluated by quantitative RT-PCR; Some *CaWRKY*s were highly expressed and up-regulated by stress treatment. Our results will provide a platform for functional identification and molecular breeding studies of WRKY genes in pepper.

## Introduction

Transcription factors are a class of proteins that regulate gene expression. They are usually composed of at least four discrete domains: a DNA binding site, a transcription activation domain, an oligomerization site and a nuclear localization signal. These domains operate together to regulate many physiological and biochemical processes, and to activate and/or repress transcription in response to endogenous and exogenous stimuli. These transcription factors facilitate the evolution and adaption of more complex developmental systems.

WRKY transcription factors are widely distributed and constitute one of the largest transcription factor families in the plant kingdom (Eulgem et al., 2000). The name is derived from the most prominent feature of these proteins. The WRKY domain is defined by the conserved amino acid sequence WRKYGQK at the N-terminus together with a C_2_H_2_- or C_2_HC-type zinc finger motif. The conserved cognate binding site of the WRKY domain in target genes is called a W box (C/TTGACT/C), which is preferentially bound by almost all WRKY transcription factors. Based on the number of WRKY domains and structure of zinc-finger motifs, WRKYs can be classified into three main groups (Eulgem et al., 2000). The WRKYs with two WRKY domains containing C_2_H_2_ zinc-finger motif belongs to Group I. The WRKYs with a single WRKY domain including a C_2_H_2_ zinc-finger motif belong to Group II, which can be further divided into five subgroups, II-a, b, c, d, and e, respectively. Group III WRKYs have single WRKY domain including a C_2_HC zinc-finger motif.

Since the first cDNA encoding a WRKY protein, *SPF*1, was cloned from sweet potato (Ishiguro and Nakamura, 1994), a large number of WRKY proteins have been identified from virtually all classes of plants, such as *Arabidopsis thaliana* (Eulgem et al., 2000; Rushton et al., 2010; Song and Gao, 2014), rice (Wu et al., 2005; Rushton et al., 2010), cucumber (Ling et al., 2011), tomato (Huang et al., 2012), soybean (Zhou et al., 2008), apple (Xu et al., 2012). Recently, as more and more plant genomes have been sequenced, genome-wide identification and functional analysis of WRKY transcription factors have been accomplished (Jiang et al., 2011, 2014; Ling et al., 2011; Huang et al., 2012; Xu et al., 2012; Zou, 2013; Ding et al., 2015; Ma et al., 2015).

Many studies about WRKY identification and functional analysis have shown that WRKY proteins play significant roles in signaling and regulation of expression during various biotic and abiotic stresses (Banerjee and Roychoudhury, 2015). In *Arabidopsis*, many *AtWRKY* genes are involved in plant defense against bacterial, fungal and viral pathogens (Li et al., 2006; Xu et al., 2006; Zheng et al., 2006, 2007; Knoth et al., 2007; Higashi et al., 2008; Kim et al., 2008; Lai et al., 2008; Pandey et al., 2010). Microarray analyses have also revealed that some of the *AtWRKY* respond strongly to various abiotic stresses, such as salinity, drought and cold (Seki et al., 2002; Kilian et al., 2007; Chen et al., 2010; Li et al., 2011). In rice, at least five *OsWRKY* genes were demonstrated to participate in the defense response against pathogens (Liu et al., 2005; Qiu et al., 2007; Shimono et al., 2007; Ramamoorthy et al., 2008), and many *OsWRKY* genes were shown to be positive and/or negative regulators of defense against abiotic stresses of heat, cold, salt or hormones (Qiu et al., 2004; Ryu et al., 2006; Liu et al., 2007). In tomato, expression of *SlWRKY*31, *SlWRKY*32, and *SlWRKY*74 were significantly up-regulated in response to drought stress, and expression of 12 *SIWRKY* genes was significantly increased under salt stress (Huang et al., 2012). In cucumber, 23 WRKY genes were differentially expressed in response to at least one abiotic stress (cold, drought or salinity; Ling et al., 2011). Three WRKY transcription factors of *Carica papaya*, TF12.199, TF807.3, and TF21.156, were up-regulated when infected by papaya ringspot virus (Pan and Jiang, 2014). The overexpression of an SA-inducible gene, *PtrWRKY*89, accelerated expression of PR protein genes and improved resistance to pathogens in transgenic poplar (Jiang et al., 2014). In *Capsicum*, a small number of WRKY genes were identified and demonstrated to display tissue-specific and induced expression patterns (Park et al., 2006; Li et al., 2008; Wang et al., 2008; Zhang, 2010). *WRKY*6, *WRKY*70, and *WRKY*-A1244 expression was induced after *R. solanacearum, P. capsici* or TMV inoculation, respectively (Li et al., 2008). *WRKY*40 played an important role in the regulation of tolerance to heat stress and to *R. solanacearum* infection (Dang et al., 2013). Overexpression of *WRKY*27 and *WRKY*58 positively and negatively regulated resistance to *R. solanacearum* infection, respectively (Wang et al., 2013; Dang et al., 2014).

Pepper is the world's second most important solanaceous vegetable after tomato, and widely cultivated and eaten both as a vegetable and as a spice. World production was more than 34 million tons (FAO, 2013; http://www.fao.org) on about 3.9 million, with China, India, and Mexico as the main growers in 2013. Because of its widespread geographical distribution and increasingly variable weather patterns are associated with climate change; pepper is vulnerable to a great number of biotic and abiotic stresses, such as pathogens, drought and high temperature, which can easily cause production drop. The WRKY family of transcription factors is one of the most important families of plant transcriptional regulators with members regulating multiple biological processes, especially in regulating defense against biotic and abiotic stresses. Thus, it is necessary to identify WRKY transcription factors, and illuminate these molecular mechanisms in regulative multiple biological processes in pepper. Based on such evidence paths to improving the resistance of pepper to stresses may be revealed. Drafts of the *Capsicum annuum* L. genome sequence were reported recently (Kim et al., 2014; Qin et al., 2014). In the current study, we searched these genome sequences to identify the WRKY genes of pepper (*CaWRKY*). Detailed analyses were then conducted, including gene classification, chromosome distribution, gene duplication, gene phylogeny, and conserved motif composition. Further, we analyzed expression of the identified 21 *CaWRKY* genes under normal growth conditions and under various abiotic and biotic stress conditions. These results will be useful for genetic improvements of agronomic traits and/or stress tolerance in pepper.

## Materials and methods

### Sequence database searches

*Arabidopsis* WRKY proteins sequences were obtained from TAIR (ftp://ftp.arabidopsis.org; Lamesch et al., 2012). The pepper annotated genome sequences were downloaded from the Pepper Genome Database (PGP, http://peppergenome.snu.ac.kr and PGD, http://peppersequence.genomics.cn; Kim et al., 2014; Qin et al., 2014). In a previous study, we identified 40 pepper WRKY proteins (*CaWRKY*1-40) which were divided into three WRKY groups (Diao et al., 2014). We used these 40 pepper WRKY proteins as query sequences for BLASTP searches against the two pepper genome databases. The sequences were selected as candidates for further study if their E value was ≤ e^−10^. Candidate sequences were confirmed for presence of WRKY domains by use of the Hmmsearch program (HMMER 3.0, http://hmmer.janelia.org/). The WRKY-like sequences confirmed by Hmmsearch in the pepper genome were in turn used reiteratively to search the pepper predicted proteins until no new sequences were found. The WRKY sequences in two different pepper genome databases were blasted using DNAMAN software, and those having same WRKY core domain with 60 amino acids were considered as one WRKY gene.

### Multiple sequence alignment, gene chromosomal location, and gene phylogenetics analysis

The 60 amino acid sequence spanning the WRKY core domain of all *CaWRKY* proteins and selected *AtWRKY* proteins [*AtWRKY*20 (At4g26640), *AtWRKY*40 (At1g80840), *AtWRKY*72 (At5g15130), *AtWRKY*50 (At5g26170), *AtWRKY*74 (At5g28650), *AtWRKY*65 (At1g29280), and *AtWRKY*54 (At2g40750)] were used to create multiple protein sequence alignments using Clustal X 2.1 with default settings (Larkin et al., 2007). The gene chromosomal locations were obtained by the pepper gene annotation giff3 file downloaded from Pepper Genome DataBase (http://peppersequence.genomics.cn). The WRKY domain boundary was defined as described (Eulgem et al., 2000). The neighbor-joining method was used to construct the phylogenetic tree based on the amino acid sequence of WRKY domains using MEGA 6.06 (Tamura et al., 2011). The parameters used in tree construction were the JTT model plus gamma-distributed rates determined by ProTest 3.0 and 1000 bootstraps (Darriba et al., 2011).

### Motif composition analysis of *Ca*WRKY proteins

The MEME 4.11.0 online program (http://meme.nbcr.net/meme/intro.html) was used for the identification of motifs in the *C. annuum* WRKY protein sequences. The optimized parameters of MEME were employed as follows: number of repetitions, any; maximum number of motifs, 20; and the optimum width of each motif, between 6 and 50 residues (Bailey et al., 2009).

### Treatments of pepper plants with various biotic and abiotic stresses and pathogen infection

Accession PI201234, highly resistant to *Phytophthora capsici*, was used throughout the study (Barksdale et al., 1984). Seedlings were grown in the greenhouse with long day condition (16-h light, 8-h dark) under a temperature of 26°C in light and 18°C in dark. Seedlings at the six true leaf stages were used for all experiment. For heat shock treatment, seedlings were subjected to 42°C. Plants were subjected to 26°C for control. For salt- and drought-stress treatments, seedlings were subjected to 300 mM NaCl and 400 mM mannitol for 24 h, respectively. Plants were subjected to sterile water for control. For pathogen infection, seedlings were infected with *Phytophthora capsici* spore suspension (10^5^ spores ml^−1^) and after were incubated under 100% relative humidity. Plants were sprayed with sterile water for control. For hormone treatments, seedlings were sprayed using a solution of salicylic acid (SA, 100 μM), methyl jasmonate (MeJA, 100 μM), or abscisic acid (ABA, 100 μM). Plants were sprayed with sterile water for control. The roots treated with drought and *Phytophthora capsici* spore suspension inoculation, and leaves treated with salt, heat shock and hormone were collected separately at 0, 3, 6, 12, and 24 h after treatment for RNA isolation.

### Real-time quantitative RT-PCR

Total RNA was isolated from the roots or leaves of PI201234 using the RNA simple total RNA kit (Takara) and was treated with DNase I (Takara) to remove any traces of genomic DNA according to the manufacturer's instructions. RNA concentration and purity were determined using a NanoDropTM spectrophotometer ND-1000 (Thermo Scientific), and RNA integrity was verified by 1% agarose gel electrophoresis.

The cDNA synthesis was carried out in a total volume of 20 μl with approximately 2 μg RNA using M-MLV Reverse Transcriptase (Promega). Real-time quantitative PCR (qRT-PCR) reaction was carried out in a total volume of 25 μl containing 12.5 μl 2 × SYBR *Premix Ex Taq*^TM^ (Takara), 1 μl (10 pmoles) of each primer, 2 μl template (10 × diluted cDNA from samples), and 8.5 μl sterile distilled water. Reaction mixtures were incubated for 30 s at 95°C, followed by 40 amplification cycles for 5 s at 95°C, and 30 s at 60°C. All reactions were carried out on 96-well reaction plates with the iQ5 machine (Bio-Rad) in triplicate. qRT-PCR analysis was performed by the comparative Ct method, which mathematically transforms the threshold cycle (Ct) into the relative expression level of genes (Perkin-Elmer User Bulletin). Primer efficiencies were calculated with software (LinRegPCR 11.0). Relative expression levels of these genes were imported to *NormFinder* analysis tools, which were used as described in their manuals. With the pepper *Actin*1 (Genebank Accession L: GQ339766) as the internal reference gene, relative gene expression values were calculated using the 2(−Ct) method (Wang et al., 2012), and data of three biological replicates were analyzed. A total of 21 *CaWRKY*s belonging to the different subgroups were randomly selected for gene expression analysis under abiotic or biotic stresses.

### Search for *cis*-acting elements in the promoters of *CaWRKY* genes

The upstream regions (500 bp) of the 20 *CaWRKY* genes which selected for qRT-RCR analysis were derived from PGP (http://peppergenome.snu.ac.kr), and were searched for regulatory elements, including W-box (binding site for the WRKY transcription factor in defense response), TATA-box (core promoter element around −30 of transcription start), CAAT-box (enhancer binding protein factors), CGTCA-motif (*cis*-acting regulatory element involved in the MeJA-responsiveness), MBS (MYB binding site involved in drought-inducibility), HSE (*cis*-acting element involved in heat stress responsiveness), TC-rich repeats (*cis*-acting element involved in the defense and stress responsiveness), SARE (*cis*-acting element involved in salicylic acid responsiveness), and ABRE (*cis*-acting element involved in the abscisic acid responsiveness) in the promoters were performed in PlantCARE (http://bioinformatics.psb.ugent.be/webtools/plantcare/html/) and PLACE database (Higo et al., 1999; Lescot et al., 2002; Guo et al., 2015).

## Results

### Identification of WRKY family members in the *Capsicum annuum* genome

A systematic analysis was performed to identify WRKY genes in the pepper genome sequences downloaded from PGP (http://peppergenome.snu.ac.kr) and PGD (http://peppersequence.genomics.cn). A total of 71 non-redundant putative WRKY genes were identified using two pepper genome databases. In previous work, forty genes (*CaWRKY*1-40) were identified (Diao et al., 2014). An additional 31 WRKY genes were identified herein and named *CaWRKY*41 to *CaWRKY*71. The annotation IDs of each *CaWRKY* in two pepper genome databases (PGP and PGD) are given in Table 1. Seven genes (*CaWRKY*56, *CaWRKY*57, *CaWRKY*60, *CaWRKY*67, *CaWRKY*69, *CaWRKY*70, and *CaWRKY*71) have only one annotation ID due to specificity of gene sequences or sequence splicing error.

**Table 1:** **WRKY transcript factor family in pepper**.

**Gene**	**Annotation ID**	**WRKY domain**			**Group**
		**Conserved heptapeptide**	**Zinc-finger type**	**Domain number**	
*CaWRKY*1	*Capana*07g002454/*Ca*07g21030	WRKYGQK/WRKYGQK	C_2_H_2_	2	I
*CaWRKY*2	*Capana*07g000181/*Ca*07g01910	WRKYGQK/WRKYGQK	C_2_H_2_	2	I
*CaWRKY*3	*Capana*11g001882/*Ca*11g03750	WRKYGQK/WRKYGQK	C_2_H_2_	2	I
*CaWRKY*4	*Capana*00g004057/*Ca*09g14010	WRKYGQK/WRKYGQK	C_2_H_2_	2	I
*CaWRKY*5	*Capana*10g001791/*Ca*10g14950	WRKYGQK/WRKYGHK	C_2_H_2_	2	I
*CaWRKY*6	*Capana*07g002350/*Ca*07g20160	WRKYGQK/WRKYGQK	C_2_H_2_	2	I
*CaWRKY*7/WRKY-c	*Capana*02g003339/*Ca*02g27910	WRKYGQK/WRKYGQK	C_2_H_2_	2	I
*CaWRKY*8/WRKY-type	*Capana*06g001506/*Ca*06g13580	WRKYGQK/WRKYGQK	C_2_H_2_	2	I
*CaWRKY*9	*Capana*07g001256/*Ca*07g10930	WRKYGQK/WRKYGQK	C_2_H_2_	2	I
*CaWRKY*42	*Capana*05g002502/*Ca*05g20090	WRKYGQK/WRKYGQK	C_2_H_2_	2	I
*CaWRKY*43	*Capana*03g003085/*Ca*03g12030	WRKYGQK/WRKYGQK	C_2_H_2_	2	I
*CaWRKY*44	*Capana*10g000205/*Ca*10g00950	WRKYGQN/WRKYGQK	C_2_H_2_	2	I
*CaWRKY*48	*Capana*10g001805/*Ca*10g14770	WRKYGQK/WRKYGQK	C_2_H_2_	2	I
*CaWRKY*58	*Capana*04g001820/*Ca*04g11710	WRKYGQK/WRKYGQK	C_2_H_2_	2	I
*CaWRKY*41/WRKY-a	*Capana*09g001251/*Ca*09g11950/ *Ca*09g11940/*Ca*09g11930	WRKYGQK/WRKYGQK	C_2_H_2_	2	I
*CaWRKY*10	*Capana*08g000683/*Ca*00g00130	WRKYGQK	C_2_H_2_	1	II (a)
*CaWRKY*11	*Capana*12g001134/*Ca*00g00230	WRKYGQK	C_2_H_2_	1	II (a)
*CaWRKY*12/WRKY-d	*Capana*03g000473/*Ca*03g32070	WRKYGQK	C_2_H_2_	1	II (a)
*CaWRKY*13	*Capana*06g001110/*Ca*00g87690	WRKYGQK	C_2_H_2_	1	II (a)
*CaWRKY*14/WRKY-* RKNIF*2	*Capana*02g002230/*Ca*02g18540	WRKYGQK	C_2_H_2_	1	II (b)
*CaWRKY*15/WRKY-6	*Capana*07g001387/*Ca*07g11490	WRKYGQK	C_2_H_2_	1	II (b)
*CaWRKY*16	*Capana*11g001631/*Ca*11g05370	WRKYGQK	C_2_H_2_	1	II (b)
*CaWRKY*50	*Capana*06g001008/*Ca*06g19170	WRKYGQK	C_2_H_2_	1	II (b)
*CaWRKY*51/*WRKY*2*-RKNIF*1	*Capana*08g001961/*Ca*00g60490	WRKYGQK	C_2_H_2_	1	II (b)
*CaWRKY*54	*Capana*02g000918/*Ca*02g08530	WRKYGQK	C_2_H_2_	1	II (b)
*CaWRKY*66	*Capana*03g001099/*Ca*00g80710	WRKYGQK	C_2_H_2_	1	II (b)
*CaWRKY*17	*Capana*07g001968/*Ca*07g15490	WRKYGQK	C_2_H_2_	1	II (c)
*CaWRKY*18/WRKY-b	*Capana*00g001033/*Ca*11g12710	WRKYGQK	C_2_H_2_	1	II (c)
*CaWRKY*19	*Capana*02g003661/*Ca*02g30960	WRKYGQK	C_2_H_2_	1	II (c)
*CaWRKY*20	*Capana*01g002803/*Ca*01g22410	WRKYGQK	C_2_H_2_	1	II (c)
*CaWRKY*21	*Capana*00g000056/*Ca*02g12180	WRKYGQK	C_2_H_2_	1	II (c)
*CaWRKY*22	*Capana*08g000429/*Ca*08g03020	WRKYGKK	C_2_H_2_	1	II (c)
*CaWRKY*23	*Capana*01g003441*/Ca*01g28150	WRKYGQK	C_2_H_2_	1	II (c)
*CaWRKY*24	*Capana*09g000676*/Ca*09g08120	WRKYGQK	C_2_H_2_	1	II (c)
*CaWRKY*45	*Capana*12g001851*/Ca*12g09140	WRKYGQK	C_2_H_2_	1	II (c)
*CaWRKY*46	*Capana*11g001905*/Ca*10g13480	WRKYGQK	C_2_H_2_	1	II (c)
*CaWRKY*47	*Capang*05g001761*/Ca*05g16170	WRKYGQK	C_2_H_2_	1	II (c)
*CaWRKY*49	*Capana*01g000165*/Ca*01g01900	WRKYGQK	C_2_H_2_	1	II (c)
*CaWRKY*64	*Capana*12g001826*/Ca*12g09290	WRKYGKK	C_2_H_2_	1	II (c)
*CaWRKY*68	*Capang*05g001761*/Ca*05g16160	WRKYGQK	C_2_H_2_	1	II (c)
*CaWRKY*25	*Capana*03g003279*/Ca*06g07080	WRKYGQK	C_2_H_2_	1	II (d)
*CaWRKY*26	*Capana*06g003072*/Ca*06g01330	WRKYGQK	C_2_H_2_	1	II (d)
*CaWRKY*27	*Capana*02g003053*/Ca*02g14640	WRKYGQK	C_2_H_2_	1	II (d)
*CaWRKY*28	*Capana*04g000568*/Ca*04g18300	WRKYGQK	C_2_H_2_	1	II (d)
*CaWRKY*52	*Capana*02g000680*/Ca*02g01800	WRKYGQK	C_2_H_2_	1	II (d)
*CaWRKY*55	*Capana*00g003083*/Ca*01g29700	WRKYGQK	C_2_H_2_	1	II (d)
*CaWRKY*56	*Ca*12g19100	WRKYGQK	C_2_H_2_	1	II (d)
*CaWRKY*60	*Ca*12g19130	WRKCGQK	C_2_H_2_	1	II (d)
*CaWRKY*67	*Ca*12g19110	WRKYGQK	C_2_H_2_	1	II (d)
*CaWRKY*29	*Capana*01g000167*/Ca*01g01920	WRKYGQK	C_2_H_2_	1	II (e)
*CaWRKY*30	*Capana*08g001012*/Ca*08g07730	WRKYGQK	C_2_H_2_	1	II (e)
*CaWRKY*31	*Capana*10g000754*/Ca*10g06160	WRKYGQK	C_2_H_2_	1	II (e)
*CaWRKY*32/WRKY-A1244	*Capana*02g001624*/Ca*02g13500	WRKYGKK	C_2_H_2_	1	II (e)
*CaWRKY*33	*Capana*02g000212*/Ca*02g03480	WRKYGQK	C_2_H_2_	1	II (e)
*CaWRKY*57	*Ca*01g23300	WRKYGQK	C_2_H_2_	1	II (e)
*CaWRKY*59	*Capana*07g001809*/Ca*07g14560	WRKYGQK	C_2_H_2_	1	II (e)
*CaWRKY*34	*Capana*10g001220*/Ca*10g06890	WRKYGQK	C_2_HC	1	III
*CaWRKY*35	*Capana*03g002072*/Ca*03g19200	WRKYGQK	C_2_HC	1	III
*CaWRKY*36/WRKY-30	*Capana*01g004472*/Ca*01g34470	WRKYGQK	C_2_HC	1	III
*CaWRKY*37	*Capang*00g001827*/Ca*01g01280	WRKYGQK	C_2_HC	1	III
*CaWRKY*38	*Capana*07g000528*/Ca*05g11500	WRKYGQK	C_2_NC	1	III
*CaWRKY*39/WRKY-70	*Capana*03g002635*/Ca*03g12230	WRKYGQK	C_2_HC	1	III
*CaWRKY*40	*Capana*08g001044*/Ca*08g08240	WRKYGQK	C_2_HC	1	III
*CaWRKY*63	*Capana*01g004471*/Ca*01g34460	WRKYGQK	C_2_HC	1	III
*CaWRKY*65	*Capang*08g001312*/Ca*01g34480	WRKYGQT	C_2_HC	1	III
*CaWRKY*71	*Capana*10g001548	WRKYGQK	C_2_HC	1	III
*CaWRKY*53	*Capana*09g001790*/Ca*09g05110	WRKYGQK	C_2_H_2_	1	NG
*CaWRKY*61	*Capana*03g002134*/Ca*03g25570	WRKYGQK	C_2_H_2_	1	NG
*CaWRKY*62	*Capana*03g001962*/Ca*03g20260	WRKYGMK	C_2_H_2_	1	NG
*CaWRKY*69	*Ca*12g19120	WRKYGQK	–	1	NG
*CaWRKY*70	*Capana*00g004852	No conserved stretch	–	–	NG

All the putative 71 WRKY genes were further analyzed to confirm the presence of the WRKY domain. As shown in Table 1, 69 *CaWRKY* genes containing complete WRKY domains were identified, and only two genes (*CaWRKY*69 and *CaWRKY*70) did not have complete domains. *CaWRKY*69 contained 288 amino acids, but did not have a zinc finger motif at its C-terminal end, and its WRKY domain contained only 38 amino acids. *CaWRKY*70 has no WRKY domain. Next, searching with WRKY in NCBI GenBank database was performed; 11 previously annotated WRKY genes (*WRKY*-a, *WRKY*-b, *WRKY*-c, *WRKY*-d, *WRKY*-type, *WRKY*-6, *WRKY*-30, *WRKY*-70, *WRKY*-RKNIF2, *WRKY*2-RKNIF1, *WRKY*-A1244) in pepper were obtained. These 11 WRKY genes were included in the 71 WRKY genes identified above, and have very few bases different with *CaWRKY* genes identified in this study (Table 1). Interestingly, we found that the sequences of *CaWRKY*41 (*Capana*09g001251) and *WRKY*-a (AAR26657) were identical; Blast analysis revealed that Ca09g11930, Ca09g 11940, and Ca09g11950 were the different parts of them.

Among the 71 *CaWRKY*s, the proteins contained from 132 aa (*CaWRKY*70) to 869 aa (*CaWRKY*9), the average length of a WRKY protein was 373 aa. The detailed information about *CaWRKY* genes, including gene loci accession number in PGP or PGD, WRKYGOK heptapeptide stretch, zinc-finger motif type, number of WRKY domains and gene classification, is listed in Table 1. The nucleotide and protein sequences of *CaWRKY* gene family are listed in Online Source 1.

### Classification of *CaWRKY*s

The most prominent structural feature of WRKY genes is the WRKY domain with a highly conserved heptapeptide stretch WRKYGQK at its N-terminus as well as a zinc-finger motif. Among these 71 *CaWRKY*s proteins identified, 15 *CaWRKY*s protein contained two WRKY domains, so a total of 85 WRKY domains were found in this study. For the two WRKY domains in the same protein, we designated the domain as the WRKY name plus N or C for the N-terminal or C-terminal domain, respectively.

The phylogenetic relationship of the 69 *CaWRKY*s proteins was examined by multiple sequence alignment of their WRKY domains containing approximately 66 amino acids except *CaWRKY*69 and *CaWRKY*70. Based on the *AtWRKY* classification and WRKY domain alignments of *CaWRKY*s (Eulgem et al., 2000), 69 *CaWRKY*s were mainly classified into three main groups (Figures 2, 3). The 15 *Ca*WRKYs with two WRKY domains were assigned to Group I according to the number of WRKY domains and the features of their zinc-finger motif of C-X_4_-C-X_22*-*23_-H -X_1_-H. *CaWRKY*s with single WRKY domain and zinc-finger-structure (C-X_4*-*5_-C-X_23_-H-X_1_-H) were assigned to Group II. The structure and phylogenetics tree of the 41 *CaWRKY* domain indicated that Group II were further divided into five subgroups: Group II-a (4), Group II-b (7), Group II-c (14), Group II-d (9), and Group II-e (7). There were only 10 *CaWRKY*s with a single WRKY domain and zine-finger structure of C-X_7_-C-X_25_-H-X_1_-C in Group III. Additionally, although *CaWRKY*53, *CaWRKY*61, and *CaWRKY*62 had a single WRKY domain and zinc-finger structure of C-X_4*-*5_-C-X_23_-H-X_1_-H, they did not fit into any groups due to the sequence divergence in their WRKY domains.

Although the WRKYGQK motif is highly conserved in WRKY transcription factors, six sequence variations were found in eight *CaWRKY*s (Table 2): WRKYGHK (*CaWRKY*5); WRKYGQN (*CaWRKY*44); WRKYGKK (*CaWRKY*22, *CaWRKY*32, *CaWRKY*64); WRKCGQK (*CaWRKY*60); WRKYGQT (*CaWRKY*65), and WRKYGMK (*CaWRKY*62). In addition, three zinc-finger form variations, C-X_7_-R-X_23_-N-X_1_-C, C-X_7_-C-X_24_-H-X_1_-C, and L-X_5_-C-X_23_-H-X_1_-H were identified in *CaWRKY*38, *CaWRKY*39, and *CaWRKY*67, respectively.

**Table 2:** **Variants of the heptapetide WRKYGQK and zinc-finger structure in WRKY domains in pepper**.

**Variants**	***CaWRKY* gene**	**Group**	**Encoding WRKY domain**
**VARIANTS OF WRKYGQK**			
WRKYGHK	*CaWRKY*5	I	Yes
WRKYGQN	*CaWRKY*44	I	Yes
WRKYGKK	*CaWRKY*22	II (c)	Yes
	*CaWRKY*32	II (e)	Yes
	*CaWRK*/64	II (c)	No
WRKCGQK	*CaWRKY*60	II (d)	Yes
WRKYGQT	*CaWRKY*65	III	Yes
WRKYGMK	*CaWRKY*62	NG	Yes
**NO CONSERVED STRETCH**			
	*CaWRKY*70	NG	No
**VARIANTS OF ZINC-FINGER FORMS**			
C-X_7_-R-X_23_-N-X_1_-C	*CaWRKY*38	III	Yes
C-X_7_-C-X_24_-H-X_1_-C	*CaWRKY*39	III	Yes
L-X_5_-V-X_23_-H-X_1_-H	*CaWRKY*67	II (d)	No

Additionally, the intron position was reported to be highly conserved in the region coding for the C-teriminal WRKY domain of Group I and the single WRKY domain of Group II and Group III members (Eulgem et al., 2000). Two major types of intron splicing were found in the conserved WRKY domains of *CaWRKY* genes, similar to WRKY domains in *AtWRKY* genes. The intron location is close to the region encoding the N-terminus of the WRKY domain in the majority of *CaWRKY* genes, while in the members of Group II-a and II-b, the position of the intron is located near the region encoding the C-teriminus of the WRKY domain (Figure 3).

### Chromosomal distribution and duplication of *CaWRKY* genes

A total of 70 *CaWRKY* genes are distributed across the 12 pepper chromosomes except *CaWRKY*70 (Figure 1). Chromosomes 1, 2, 3, and 7 contain relatively more *CaWRKY* genes, with 10, 9, 8, and 8 genes, respectively. Chromosomes 4 and 5 contain relatively few *CaWRKY* genes, with only 2 and 3 genes, respectively. Nine out of 71 (12.7%) *CaWRKY* genes are located on chromosome 2, while the sequenced size of chromosome 2 (156.37 M) only accounts for approximately 4.87% of the assembled pepper genome (3.13 G), *CaWRKY* genes were enriched in chromosome 2.

**Figure 1:** **Mapping of the WRKY gene family on *Capsicum annuum* L. chromosomes**. The size of a chromosome is indicated by its relative length. Tandemly duplicated genes are indicated in red.

**Figure 2:** **Unrooted phylogenetic tree representing relationships among WRKY domains of pepper and *Arabidopsis.*** The amino acid sequences of the WRKY domain of all *CaWRKY* and *AtWRKY* proteins were aligned with Clustal W and the phylogenetics tree was constructed using the neighbor-joining method in MEGA 6.0. Group I proteins with the suffix “N” or “C” indicates the N-terminal WRKY domains or the C-terminal WRKY domains. The red arcs indicate different groups or subgroups of WRKY domains.

**Figure 3:** **Alignment of multiple *CaWRKY* and selected *AtWRKY* domain amino acid sequences**. Alignment was performed using DNAman. The suffix “N” or “C” indicates the N-terminal WRKY domain or the C-terminal WRKY domain, respectively, of a specific WRKY protein. The amino acids forming the zinc-finger motif are highlighted in red. The conserved WRKY amino acid signature is highlighted in green, and gaps are marked with dashes. The position of a conserved intron is indicated by an arrowhead.

Subsequently, we further determined the tandem duplications of *CaWRKY* genes along the 12 pepper chromosomes. The tandemly duplicated genes were defined as an array of two or more homologous genes within a 100-kb range distance. As shown in Figure 1, four *CaWRKY* gene clusters (genes labeled in red) containing 11 tandemly duplicated genes were identified on chromosomes 1, 5, and 12.

### Motif composition analysis of *CaWRKY* proteins

The conserved motifs of WRKY family proteins in pepper and *Arabidopsis* were investigated using MEME version 4.11.0 online software (http://meme.nbcr.net/meme/cgi-bin/meme.cgi) to better understand the similarity and diversity of motif compositions. Twenty distinct motifs were identified, and a schematic overview of the identified motifs is provided in Figure 4 (Online Source 2). Among the 20 motifs, motifs 1, 2, and 3 together comprised the C-terminal WRKY domain, and motif 4 and motif 6 comprised the N-terminal WRKY domain in pepper. As displayed schematically in Figure 4, one or more conserved motifs outside of the WRKY domain motif can be detected in one of the pepper WRKY proteins. When comparing the motifs of *CaWRKY* and *AtWRKY* proteins, they shared the most of conserved motifs, and no motif was specific to pepper or *Arabidopsis*.

**Figure 4:** **Alignment of multiple *CaWRKY* and selected *AtWRKY* domain amino acid sequences schematic diagram of amino acid motifs of *CaWRKY* and *AtWRKY* protein groups or subgroups**. Motif analysis was performed using Meme 4.11.0 software as described in the methods. The WRKY proteins are listed on the left. The different-colored boxes represent different motifs and their position in each WRKY sequence. The sequences of key motifs (motifl, motif2, motif2, and motif4) were shown on the bottom right of Figure. A detailed motif introduction for all *CaWRKY* protein is shown in Online Source 2.

As shown in Figure 4, most *CaWRKY* members in the same group or subgroup share common motif compositions. There have not motifs shared by different groups except C-terminal WRKY domain which containing motifs 1, 2, and 3. Motif 4, motif 6 and motif 11 are unique motifs in Group I. Motif 10 is unique in Group II-b. Motif 12 and motif 16 are unique in Group III. Group II-d contains four unique motif, motif 13, 14, 15, and 19. We found that two motifs (motif 15 and motif 19) always occurred in four WRKY genes (*CaWRKY*56, *CaWRKY*60, *CaWRKY*67, and *CaWRKY*69). It is noteworthy that the characterized motif compositions allow Group II-d members in pepper to be divided into distinct subclasses. Interestingly, *CaWRKY*69 was not associated with any group due to lack of the whole WRKY domain, but it did contain five motifs (motif 13, motif 14, motif 15, and motif 19) which only existed in Group II-d, so we speculated that *CaWRKY*69 belongs to Group II-d. Group II-a and Group II-b are two close subgroups in the phylogenetics tree, motif 7 and motif 9 are frequent in the vast majority of the members of these two subgroups. Some motifs occurred in only a few *CaWRKY*s genes. For example, motif 18 was only present in *CaWRKY*5, *CaWRKY*43 and *CaWRKY*48.

### Expression patterns of *CaWRKY* genes under normal growth conditions and various abiotic and biotic stress conditions

We analyzed the expression patterns of 21 *CaWRKY*s belonging to the different subgroups under normal growth conditions and various abiotic and biotic stress conditions using real-time quantitative RT-PCR. Seven stress conditions (salt, heat, drought, *Phytophthora capsici* inoculation, SA, MeJA, and ABA) were conducted. The gene-specific primers of 21 selected *CaWRKY* genes under abiotic and biotic stress conditions are listed in Online Source 3.

As shown in Figure 5 the vast majority of the *CaWRKY* genes selected were expressed in plants grown under normal growth or treatment conditions, and the *CaWRKY* genes displayed distinct expression patterns in response to different stress treatments. Expression levels of the majority of the *CaWRKY* genes were affected within 24 h after treatment. Generally, changes of expression levels were dramatic for four genes (*CaWRKY*8, *CaWRKY*12, *CaWRKY*14, and *CaWRKY*18). However, we also found some *CaWRKY* that were not expressed during stress treatment. For example, *CaWRKY*10 did not show any detectable expression in two different tissues under different stress treatment except under drought and SA treatment, and *CaWRKY*38 did not show any detectable expression under different stress treatments but did respond to treatment with MeJA and ABA.

**Figure 5:** **Heat map showing *CaWRKY* genes expression pattern in pepper under seven different stresses**. Leaves or roots of seedlings (six true leaves) are used to test the changes of *CaWRKY* genes expression level at different timepoints (0, 3, 6, 12, and 24 h) with Salt, Heat shock, Drought, *Phytophtora capsici*, SA, MeJA, and ABA treatment. *Action*1 is used as an internal control. qRT-PCR data are shown relative to 0 h. The relative expression leves were calculated using the 2(−Ct) method. The heat man was created using R.

Under salt treatment, five genes (*CaWRKY*10, *CaWRKY*19, *CaWRKY*30, *CaWRKY*34, and *CaWRKY*38) did not show detectable expression for control or treatment. Expression of *CaWRKY*12, *CaWRKY*16, *CaWRKY*22, and *CaWRKY*32 were significantly up-regulated in response to treatment (Figure 5, genes labeled in red or dark green), while the expression of *CaWRKY*7 was down-regulated.

Under heat shock treatment, as shown in Figure 5, Expressions of four genes (*CaWRKY*8, *CaWRKY*12, *CaWRKY*14, and *CaWRKY*28) were up-regulated and another three genes (*CaWRKY*7, *CaWRKY*11, and *CaWRKY*16) were down-regulated. *CaWRKY*10, *CaWRKY*19, *CaWRKY*30, *CaWRKY*34, and *CaWRKY*38 were also not expressed for control or treated plants (Figure 5).

Under drought treatment, five genes (*CaWRKY*8, *CaWRKY*12, *CaWRKY*14, *CaWRKY*16, and *CaWRKY*18) were expressed with relatively higher intensities, and showed significant up-regulated, *CaWRKY*22, and *CaWRKY*26 were expressed with relatively lower expression intensities (Figure 5). The expression of five genes (*CaWRKY*2, *CaWRKY*11, *CaWRKY*19 *CaWRKY*24, and *CaWRKY*26) was down-regulated; and the expression of *CaWRKY*1 and *CaWRKY*3 had no significant change. Three genes (*CaWRKY*30, *CaWRKY*34, and *CaWRKY*38) did not show detectable expression for control or treatment, *CaWRKY*10 was expressed at 12 h after treatment (Figure 5).

As shown in Figure 5, *CaWRKY*34 and *CaWRKY*38 did not have detectable expression for control or treatment, and three genes (*CaWRKY*7, *CaWRKY*19, and *CaWRKY*22) were expressed with relatively lower expression intensities under *Phytophtora capsici* inoculation. The expressions of three genes (*CaWRKY*8, *CaWRKY*18, and *CaWRKY*32) and six genes (*CaWRKY*2, *CaWRKY*7, *CaWRKY*11, *CaWRKY*19, *CaWRKY*24, and *CaWRKY*26) were respectively up-regulated and down-regulated. Generally speaking, these 21 selected *CaWRKY* have not shown distinct change after *Phytophtora capsici* inoculation.

Some of the *CaWRKY* genes responded similarity to the three different hormone treatments observed in Figure 5. For example, under SA treatment, two groups of three genes each, the expression of *CaWRKY*8, *CaWRKY*14, *CaWRKY*30 and *CaWRKY*7, *CaWRKY*11, *CaWRKY*24 were up-regulated and down-regulated, respectively. Likewise, the expression of *CaWRKY*8, *CaWRKY*14 and *CaWRKY*30 were also up-regulated under MeJA and ABA treatments (Figure 5). Under MeJA and ABA treatment, the genes with lower expression intensities were still *CaWRKY*7, *CaWRKY*11, and *CaWRKY*24, and down-regulated. As shown in Figure 5, strong response to SA in *CaWRKY*10 and *CaWRKY*34 was observed after 6 h treatment, *CaWRKY*34 and *CaWRKY*38 shown detectable expression after MeJA and ABA treatment.

### Analysis of stress-related *cis*-elements in the *CaWRKY* promoters

For further understand the possible regulation mechanism of *CaWRKY* genes in the abiotic or biotic stresses response of pepper, we scanned the *cis*-elements involving in the activation of defense related genes in the promoter regions of *CaWRKY*. The promoter regions (−500 bp upstream of the translation start site) of a total of 20 *CaWRKY* genes which were applied for qRT-PCR analyzing except *CaWRKY*11 from PGP were used. Predicted *cis*-elements in the promoter regions of 20 *CaWRKY* genes were shown in Figure 6. W-box element was found in four selected promoter regions of *CaWRKY*8, *CaWRKY*14, *CaWRKY*24, and *CaWRKY*34, respectively. One to nine TATA-box elements were found in the promoter regions of 20 genes, respectively, the number of TATA-box elements in the promoter regions of *CaWRKY* was the maximum in *CaWRKY*10 and minimum in *CaWRKY*24, respectively. One to 8 CAAT-box elements were also found in promoter regions of 19 genes except *CaWRKY*24, respectively, in which the number of CAAT-box elements in the promoter region of *CaWRKY*28 and *CaWRKY*32 was the maximum (8). In addition, other stress-related *cis*-elements were detected, including CGTCA-motifs in four genes (*CaWRKY*1, *CaWRKY*3, *CaWRKY*16, and *CaWRKY*18), MBS elements in five genes (*CaWRKY*1, *CaWRKY*7, *CaWRKY*8, *CaWRKY*18, and *CaWRKY*22), HSE elements in four genes (*CaWRKY*8, *CaWRKY*12, *CaWRKY*19, and *CaWRKY*32), TC-rich repeats in five genes (*CaWRKY*9, *CaWRKY*18, *CaWRKY*19, *CaWRKY*24, and *CaWRKY*26), SARE element in *CaWRKY*3 and ABRE elements in *CaWRKY*12 and *CaWRKY*14, respectively.

**Figure 6:** **Predicted *cis*-elements in the promoter regions of *CaWRKY* genes**. Promoter sequences (−500 bp) for 20 *CaWRKY* genes (promoter regions of *CaWRKYll* was absent) were analyzed. The name of the promotes of *CaWRKY* genes are shown on the left side of the figure. The number at the bottom indicates the number of the nucleotides to the translation initiation codon, ATG. The green dovetail for the TATA-box elements, the red triangles for CAAT-box element, the yellow square for the W-box elements, the purple five-pointed star for CGTCA-motif, the black diamond for MBS, the dark green pentagon for the HSEs, the orange oval for TC-rich repeats, the blue pentagon for SARE, the pink concentrically for abscisic acid responsiveness ABRE.

## Discussion

### WRKY gene expansion and evolution in pepper

In this study, 71 WRKY genes were identified in pepper using two pepper genome databases (PGP, http://peppergenome.snu.ac.kr and PGD, http://peppersequence.genomics.cn). The WRKY gene family has 72, 109, and 81 members in *Arabidopsis*, rice and tomato, respectively. Compared with *Arabidopsis* (genome size 125 Mb), rice (480 Mb), and tomato (781 Mb), in pepper (3.13 Gb), the number of the WRKY family is comparatively very small. Considering subgroups of WRKY genes among *Arabidopsis*, rice and tomato, we found that the number of Group II(e) *CaWRKY* genes (7) was much less than that for tomato (17) and rice (11), and the number of Group III *CaWRKY* genes (10) was also much less than those of rice (36) and *Arabidopsis* (14). In this regard, pepper appears similar to cucumber. Ling et al. (2011) found the number of Group III *CsWRKY* genes was much less than that for rice (36) and *Arabidopsis* (14), and suspected that *CsWRKY*s, especially Group III *CsWRKY* genes, were underrepresented in their analysis. Complete and accurate annotation of genes is an essential starting point for further evolutionary and functional studies of this gene family. In our study, we identified a total of 71 *CaWRKY* genes after using 40 pepper WRKY proteins as query sequences and Blastp searches against the two pepper genome databases (PGP and PGD). The sequences of each WRKY gene in the two pepper genome databases were nearly identical. In addition, 11 known *CaWRKY* genes in NCBI were used to evaluate the presence of additional WRKY proteins. The results showed that certain *CaWRKY* genes are highly homologous with some *CaWRKY* genes identified in this study. Interestingly, we found that Ca09g11930, Ca09g11940, and Ca09g11950 were the different parts of *WRKY*-a (AAR26657). Therefore, we believe that *CaWRKY* genes were not underrepresented in our study.

Gene duplication events are important in the rapid expansion and evolution of gene families (Cannon et al., 2004). Tandem gene duplication of WRKY transcription factors has been observed in many plant species, such as *Arabidopsis*, rice, cucumber and tomato, etc. It was also observed in our investigation, and 15.5% (11/71) *CaWRKY* genes were found to evolve from tandem gene duplication (Figure 1). Therefore, tandem gene duplication may have played an important role in WRKY gene family expansion in pepper. Tandem gene duplication of WRKY genes was mainly associated with Group III in *Arabidopsis* and rice, and with Group II(e) in tomato. The present analysis revealed that gene expansion also occurred in Group III in pepper, evidenced by three *CaWRKY* genes (*CaWRKY*36, *CaWRKY*63, and *CaWRKY*65) clustered as middle branching members of Group III. This notion was further supported by similar WRKY domains found in other *Solanaceous* species including potato (XP_006352253.1, XP_006343875.1, and XP_006339686.1), tomato (XP_004244630.1 and XP_004 245530.1) and tobacco (AII99839.1 and AAF61864.1). Meanwhile, the chromosomal distribution of *CaWRKY* genes revealed that a tandem gene duplication may have occurred in Group II(d) in pepper. These three genes (*CaWRKY*56, *CaWRKY*60, *CaWRKY*67) were clustered as early branching members of Group II(d), the homology of these three genes was not high and the identity was only 72%. Thus, we suspect that the gene expansion has not occurred in Group II(d). The use of three WRKY proteins as query sequences for Blastp searches in the NCBI database revealed no similar WRKY domains in other *Solanaceae* species.

### *CaWRKY* proteins play important roles in various biological processes

Accumulating evidence suggests the WRKY transcription factors are involved in many plant processes including plant development, responses to biotic and abiotic stresses, and play an important role in plant defense responses. Some of the pepper WRKY genes displayed tissue specific and induced expression patterns in prior research (Park et al., 2006; Li et al., 2008; Wang et al., 2008; Zhang, 2010). The expression of *CaRKNIF*1 gene was tissue specific, and with relative higher expression in roots and young leaves. It also can be induced by *R. solanacearum, P. capsici* and TMV but not by *M. incognita* (Zhang, 2010). *WRKY*6, *WRKY*70 and *WRKY*-A1244 showed induced expression patterns under *R. solanacearum, P. capsici* and TMV inoculation, respectively (Li et al., 2008). *WRKY*-a can be induced during hypersensitive response to tobacco mosaic virus and *Xanthomonas campestris* (Park et al., 2006).

To obtain more insights into the expression patterns and putative functions of *CaWRKY* genes, 21 *CaWRKY* genes belonging to different subgroups were random selected, and their expressions in response to seven different stresses were evaluated by real-time quantitative RT-PCR analysis in this study. Some of the chosen *CaWRKY* genes have high identities with known WRKY genes in pepper, *SIWRKY* genes in tomato and *AtWRKY* in *Arabidopsis*. For example, *CaWRKY*12 has 99 and 98% identity with *SIWRKY*39 and *AtWRKY*40, respectively. *CaWRKY*18 has 99 and 98% identity with *SIWRKY*75 and *AtWRKY*75, respectively. In *Arabidopsis, AtWRKY*40 was demonstrated as a negative regulator in the defense against *Pseudomonas syringae* and the fungal pathogen *Golovinomyces orontii*, respectively. *AtWRKY*75 RNAi transgenic lines were more sensitive to low Pi stress compared to wild-type *Arabidopsis* seedlings (Dong et al., 2003). In tomato, *SIWRKY*39 showed significant up-regulated induced expression patterns under drought, salt and invasion of pathogen, elicitor, and virus (Huang et al., 2012). In our study, *CaWRKY*12 and *CaWRKY*18 were expressed with relatively high intensities, and were also significantly up-regulated by the seven stress treatments utilized in this research. These results suggest that these WRKY genes may have similar expression and function as those in tomato and pepper.

*CaWRKY*3 has 99 and 98% identity with *CaRKNIF*1 in pepper and *SIWRKY*4 in tomato, respectively. *CaRKNIF*1 can be induced by *R. solanacearum, P. capsici* and TMV but not by *M. incognita*. *SIWRKY*4 was induced by drought, salt and pathogen invasion. The expression of *CaWRKY*3 was up-regulated by heat shock, MeJA and ABA. Taken together, these observations suggested that *CaWRKY*3 can be induced not only by pathogens, but also by other biotic stresses.

Pepper WRKY genes orthologous to those in *Arabidopsis* and tomato include *CaWRKY*3, *CaWRKY*7, *CaWRKY*8, *CaWRKY*12, *CaWRKY*14, *CaWRKY*18, *CaWRKY*21, *CaWRKY*22, and *CaWRKY*32, all of them showed significant induction under stress. Meanwhile, we also found an interesting phenomenon when analysis correlation between gene expression level and W-box existing in the promoter region W-box element was presented in the promoter regions of the *CaWRKY*8 and *CaWRKY*14, which two genes showed a significantly up-regulated by stresses treatment applied in this study. It is well known that WRKY transcription factors are activated under abiotic or biotic stresses, and bind the W-box element of the promoters of the function genes to regulate the expression of downstream function genes. Thus, we predicted that *CaWRKY*8 and *CaWRKY*14 were activated by other *CaWRKY* transcription factors due to the high expression level under stresses treatment. We will verify function characters of these two genes in future work. These results imply that these members might be regulators of responses to various biotic and abiotic stresses. To date, only three *CaWRKY* genes have been functionally characterized, while the biological and cellular functions of most *CaWRKY* genes remain largely unknown. The current investigation demonstrates a number of *CaWRKY* genes that might be involved in stress defense, and provides clues for the selection of candidate genes, especially *CaWRKY*8 and *CaWRKY*14, for further studies.

## Author contributions

SW and JS designed the project, and did literature research; WD performed the main part of data acquisition, statistical analysis, and manuscript editing; JL and BP performed the main part of experimental studies; GG and GW participated in the research and analyzed the data. All authors read and approved the final manuscript.

### Conflict of interest statement

The authors declare that the research was conducted in the absence of any commercial or financial relationships that could be construed as a potential conflict of interest.
